RETRACTED

# Serum Expression Level of MicroRNA-122 and Its Significance in Patients with Hepatitis B Virus Infection

**DOI:** 10.1155/2022/8430276

**Published:** 2022-02-24

**Authors:** Qingqing Fang, Wei Chen, Yourong Jian, Yu Li, Wei Lian, Hongyu Wan, Shiyao Chen, Feng Li, Ying Chen

**Affiliations:** ^1^Department of Gastroenterology, Minhang Hospital, Fudan University, Shanghai 201199, China; ^2^Department of Gastroenterology, Zhongshan Hospital, Fudan University, Shanghai 200032, China

## Abstract

**Objectives:**

To analyze the expression of miR-122 and evaluate its significance in patients with HBV infection in different phases.

**Methods:**

Eleven chronic hepatitis B (CHB), 26 hepatitis B virus (HBV)-induced cirrhosis, 16 HBV-associated hepatocellular carcinoma (HCC) patients and 10 healthy control cases were enrolled. The serum levels of miR-122 were detected by RT-PCR and compared between healthy individuals and CHB at different stages.

**Results:**

Compared with healthy control cases, serum miR-122 levels were markedly increased in HBV infection cases (AUC = 0.795, *P*=0.002). In the CHB group, miR-122 levels were positively associated with albumin levels (*P* < 0.05) but had no significant associations with alanine aminotransferase (ALT) and aspartate aminotransferase (AST) (*P* > 0.05). In the cirrhosis group, miR-122 expression was remarkably lower in the Child C group in comparison with the Child A group (*P*=0.025). At the same time, miR-122 amounts had a negative correlation with HVPG (*P* < 0.05). In the HCC group, miR-122 amounts were negatively associated with alkaline phosphatase (AKP) and alpha-fetoprotein (AFP) (*P* < 0.05). Serum miR-122 amounts in 3 patients who died were lower than the survival group (5.520 ± 0.522 vs. 5.860 ± 1.183, *P* > 0.05).

**Conclusion:**

Serum miR-122 can be leveraged to screen patients with HBV infection. In HBV sufferers, the serum miR-122 expression level is related to liver disease progression, hence making it an underlying molecular biomarker for predicting the development of CHB.

## 1. Introduction

More than 250 million individuals globally have chronic HBV infection [1]. Persistent HBV infection might induce hepatic damage and develop into advanced hepatic pathologies. Approximately 3%–6% hepatic sclerosis cases may progress to primary HCC [2]. Hence, HBV patients with worsening liver function and decompensating liver cirrhosis should be imperatively assessed at the disease early stage.

HBV replication is modulated by various host factors, including miRNAs. miRNAs are remarkably conserved small ncRNAs that simultaneously regulate physiological and pathological functions in the liver. Changes in the expression of miRNAs are related to hepatic metabolic disorders, hepatic damages, hepatic fibrosis, and tumor progression, which make miRNAs appealing targets for the diagnoses and treatment of hepatic diseases [3].

RETRACTED

Research has revealed that an overall 277 miRNAs are expressed in the liver, of which microRNA-122 (miR-122) is considered one of the most potent miRNAs [4, 5]. MiR-122 was shown to decrease HBV DNA levels by downregulating cyclin G1, a negative modulator of p53 [6]. Moreover, miR-122 participates in the intricate signal transmission network in BP involved in hepatic development and differentiation, liver lipidic metabolism, stress reactions, and HCC [7–10]. In addition, miR-122 is related to the phase and seriousness of the infection. This correlation might help measure therapeutic effects [11–13].

The present work aimed to assess miR-122 expression in diverse phases of CHB infection and to examine its significance.

## 2. Materials and Methods

### 2.1. Patients

This trial enrolled CHB, hepatitis B-induced sclerosis, and hepatitis B-related HCC patients in the Department of Gastroenterology, Minhang Hospital, Fudan University, from June 2020 to June 2021.

Inclusion criteria were as follows: (1) control group, healthy subjects; (2) CHB group, meeting the diagnostic criteria for chronic hepatitis [14]; (3) hepatitis B cirrhosis group, HBV history, and meeting the diagnostic criteria of the guidelines for diagnosing and treating hepatic sclerosis [15]; and (4) HBV-associated HCC group, HBV history combined with clinical imaging, laboratory indicators, and/or liver biopsy indicating HCC.

Exclusion criteria were as follows: (1) liver damage induced by other causes, including HCV infection, drug intake, drinking quantity, and AIH; (2) severe heart, lung, kidney, and/or systemic diseases; (3) liver cirrhosis and liver cancer caused by other chronic liver diseases; and (4) combination with other malignant tumors. All eligible patients and healthy controls provided written informed consent, and all assays were accepted by the Ethical Board of Minhang Hospital affiliated to Fudan University (batch number: 006-01K).

### 2.2. Serum Sample Collection

Peripheral blood samples (*n* = 63) were collected and centrifuged at 3000 g for 10 minutes at ambient temperature. The resulting supernatants were further subjected to centrifugation for 10 minutes at 4°C. Then, serum was immediately kept at −80°C until utilization.

### 2.3. Methods

#### 2.3.1. Determination of miRNA-122 Levels in Serum

The PerfectStart^TM^ Green qPCR SuperMix kit was employed to assess miRNA-122 levels on a LightCycler® 480 II fluorescent quantitation PCR equipment (Roche, Switzerland). The reaction included 2× PerfectStart^TM^ Green qPCR SuperMix (5 *μ*l), 10 *μ*M Universal primer (0.2 *μ*l), 10 *μ*M microRNA-specific primer (0.2 *μ*l), cDNA (1 *μ*l), and nuclease-free water (3.6 *μ*l). Amplification was carried out at 94°C (30 s), followed by 45 cycles of 94°C (5 s) and 60°C (30 s). After the last cycle, a melting curve was utilized to detect product specificity: the temperature was increased from 60°C to 97°C, and fluorescence was recorded 5 times per centigrade. miRNA-122 expression was computed by the 2^−∆∆*Ct*^ method.

RETRACTED

#### 2.3.2. Blood Routine, Biochemical Function, and AFP Measurement

Automatic routine biochemical and immune analyzers were utilized to measure blood routine, liver and kidney function, and AFP.

#### 2.3.3. HVPG Measurement

The hepatic vein wedge pressure and free pressure were measured by jugular vein catheterization, and the difference between the two was HVPG [16].

### 2.4. Statistics

SPSS 23.0 program was leveraged to assess the data. The data were described as *x* ± *s*, and one-way ANOVA was utilized for multigroup comparisons. The *t*-test was performed for group pair comparisons. Categorical variables were compared by the *χ*^2^ test. Pearson correlation analysis was utilized for classification, rank, or non-normally distributed continuous data. Spearman correlation analysis was utilized for normally distributed continuous data. *P* < 0.05 was considered statistically significant.

## 3. Results

### 3.1. Baseline Patient Characteristics

This study enrolled 10 healthy controls, 11 CHB, and 26 hepatic sclerosis cases. There were 10 Child A, 11 Child B, 5 Child C, and 16 HCC cases. No remarkable differences in gender and age were found among these four groups of patients. In terms of HGB, WBC count, Cr, TB, DB, AKP, Alb, and AFP, there were significant differences (Table 1). The data are detailed in Table 1.

### 3.2. Serum miR-122 Amounts in Healthy Controls and Cases with Different Stages of HBV Infection

In contrast to the healthy control cases, the expression levels of miR-122 were increased significantly in the CHB, HBV-related cirrhosis, and HCC groups (Figure 1; all *P* < 0.05). Among the infected patients, the highest miR-122 amounts were detected in the CHB group (*P* < 0.05). There were no remarkable diversities between the cirrhosis and HCC groups in terms of miR-122 levels (*P*=0.878).

### 3.3. Significance of Serum miR-122 Expressing in Chronic Hepatitis B

ROC curves were generated for assessing the diagnostic efficacy of serum miR-122 in CHB. Serum miR-122 expression displayed a great diagnostic value for HBV infection (Figure 2(a); AUC = 0.795, *P*=0.002). Therefore, serum miR-122 was expected to be effective in screening patients with HBV infection. Meanwhile, in the CHB group, serum miR-122 was significantly associated with albumin content (Figure 2(b), *P*=0.030) but showed no associations with ALT and AST (both *P* > 0.05).

RETRACTED

### 3.4. Significance of Serum miR-122 Expression in Cirrhosis

In the hepatic sclerosis group, serum miR-122 amounts in cases with distinct Child–Pugh scores were different, which were higher in Child A cases than Child C cases (Figure 3(a), *P* < 0.05). More importantly, serum miR-122 amounts were negatively associated with HVPG (Figure 3(b), *P*=0.037). Serum miR-122 amounts in cases with HVPG ≤ 10 and HVPG > 10 were 6.741 ± 1.177 and 5.788 ± 0.838, respectively (Figure 3(c), *P*=0.062). Therefore, miR-122 may be an effective index for predicting further decompensation of liver cirrhosis and aggravation of portal hypertension.

### 3.5. Significance of Serum miR-122 Expression in Hepatocellular Carcinoma

The associations of clinical indexes with miR-122 in 16 serum specimens in the HCC group were assessed. As shown in Figures 4(a) and 4(b), serum AKP and AFP were increased, while serum miR-122 was reduced, indicating negative correlations (*P*=0.035 and *P*=0.029).

## 4. Discussion

Timely diagnosis of persistent viral hepatitis is vital for treating and preventing hepatitis, which can also help inhibit disease progression and reduce disease spread in the population to a large extent [17, 18]. In a meta-analysis [19], miR-122 was found to exhibit sensitivity and sensitivity of 0.92 and 0.84 in the diagnosis of chronic viral hepatitis, respectively; only 10% of negative results were false negatives. As shown above, miR-122 could detect CHB with an AUC of 0.795 (*P*=0.002). Because of insufficient samples in this study, we could not verify the results in an external cohort. Consequently, the clinical significance of miR-122 application in diagnosis deserves further investigation.

A few studies [20–22] have examined the role of microRNAs in HBV infection. The correlation between HBV duplication and miR-122 has been explored as well. After exposure of hepatocytes to HBV, inflammation leads to increased cell necrosis and apoptosis, and massive miR-122 amounts are released into the circulation [23]. After released by damaged hepatocytes, the microRNAs cumulate persistently and reach a greater level. HBV DNAs, as the most direct and dependable indicator of virus duplication, is capable of straightly reflecting the virus and the infection ability in vivo. As shown above, serum miR-122 was remarkably increased in CHB cases compared with control individuals. There was a report that serum miR-122 amounts are tightly associated with HBV [24]. Serum miR-122 levels are elevated in HBV patients. Therefore, miR-122 might become a sensitive marker reflecting hepatitis activity in HBV cases.

RETRACTED

In different phases of HBV infection, albumin indexes of patients were positively correlated with miR-122 levels in the CHB group, as shown above. Albumin from the liver has functions such as immune regulation and antioxidation. It was shown that miR-122 exerts negative modulatory effects on HBV replication [25, 26]. In terms of HBV modulation, Chen et al. [27] have revealed that miR-122 is capable of binding to the remarkably conservative area of a bicistronic mRNA referred to as HBV pregenomic RNA, which has been discovered to be capable of encoding the HBV polymerase and core protein. Hence, it eventually induces the suppression of HBV genetic expression and duplication. Therefore, the decrease of serum miR-122 weakens the inhibitory effect of HBV DNA replication, thereby aggravating the injury and causing a decrease in albumin. In the liver cancer group, the expression of miR-122 in patients was related to AKP indicators in a negative way. AKP is often associated with impaired liver functions. In two other studies [10, 28], it was found that miR-122 amounts in CHB are negatively correlated with HBV DNA, ALT, and HBsAg levels. Therefore, we speculate that miR-122 may be associated with the severity of hepatocyte damage. Briefly, the lower the miR-122 expression, the severer the hepatocyte damage and the worse the prognosis.

After hepatitis B infection, with disease progression, miR-122 levels gradually decreased. This study demonstrated miR-122 amounts were highest in the CHB group but lower in the liver cancer group in comparison with the liver cirrhosis group, although statistical significance was not reached. These lower serum miRNA levels in patients with more advanced illness may be secondary to their decreased excretion because of the absence of functional liver cells instead of their elevated releasing from damaged liver cells in earlier phases of hepatic illnesses [29–31]. Those diversities may reveal that miR-122 might be one of the stimulative factors in the development of HBV-triggered illnesses. In the cirrhosis group, we found that miR-122 expression was related to the Child–Pugh class. Cirrhosis is a progressive disease, and each stage has distinct clinical and prognostic features. Studies have shown miR-122 affects HBV replication in vitro and is remarkably related to HBV-associated hepatic sclerosis [32]. MicroRNAs participate primarily in the response to low oxygen by regulating key genes participating in apoptosis, including BCL2 and XIAP. Hypoxia is vital for the development of sclerosis because it activates revascularization, suppresses cellular proliferative factors, and induces fibrogenic activities, fostering gradual portal pressure elevation and hyperdynamic circulation [33, 34]. The antifibrotic disorders of miRNAs induce the onset of hepatic sclerosis in CHB cases [35], and the decreased expression of miR-122 weakens the inhibitory effect on liver fibrosis, thereby aggravating the occurrence of liver cirrhosis, which corroborates this study. Interestingly, in the cirrhosis group, miR-122 was negatively associated with HVPG, as shown above. The serum miR-122 of 4 patients with HVPG < 10 mmHg was higher than 21 patients with HVPG > 10 mmHg. HVPG ≥ 10 mmHg is the gold standard for the diagnosis of CSPH [36], and an independent risk factor for rebleeding in hepatic sclerosis [37]. Here, we found that the lower the miR-122 expression, the higher the portal pressure, the greater the risk of portal hypertension-related complicating diseases such as hemorrhage, and the worse the prognosis. However, HVPG can only be assessed by invasive methods that require the proficiency of doctors in major hospitals. miRNA-122 is expected to become a new noninvasive biomarker that could be used as an alternative to HVPG. Cirrhosis is a progressive disease, each stage of which exhibits distinct clinical and prognostic features. As the disease progressed, miR-122 was downregulated in this study. Therefore, we speculate that miR-122 is associated with the development of hepatic illnesses.

RETRACTED

In addition, miR-122 has been discovered to participate in the process of hepatic cancer. One discovered the causal link beneath the progression of hepatic carcinoma is the variant of cancer inhibitor genes triggered by the overexpression of apolipoprotein B mRNA-editing enzyme catalytic subunit 2 (APOBEC2) in liver cells. The role of HBV in APOBEC2 was demonstrated through the downregulation of cellular miR-122, which promotes carcinogenesis in hepatocytes [38]. miR-122 can also regulate the activity and stability of the p53 protein by modulating regulatory proteins of the cell cycle, thereby inhibiting tumor metastasis [39]. The low expression of miR-122 can regulate the onset and progression of cancer through a variety of pathways and can be utilized as a biomarker for early hepatic carcinoma diagnoses [40]. The expression of miR-122 is high in mature hepatocytes but remarkably downregulated in HCC. This downregulation is tightly associated with liver carcinogenesis, unsatisfactory prognosis, and metastasis in HCC [41]. In the latter study, tumor-free survival time in HCC cases who exhibited high miR-122 expression was remarkably longer compared with the remaining ones, suggesting miR-122 is tightly associated with prognosis in hepatic carcinoma. In this report, serum miR-122 amounts were lowest in the liver cancer group and were correlated with AFP, whereas the ROC curve results indicated that the sensitiveness and specificness of miR-122 for the diagnosis of liver cancer were not satisfactory. This might be due to the insufficient samples herein. Overall, miR-122 is expected to become an effective biomarker for the early diagnosis of liver cancer. Our team also found that 4 of the 16 patients in the liver cancer group died, due to liver cancer combined with gastrointestinal bleeding (*n* = 1), liver cancer combined with liver failure (*n* = 2), and cardiac insufficiency (*n* = 1; this patient was excluded). The serum miR-122 amounts of three patients in the death group were 5.520 ± 0.522, which were lower than 5.860 ± 1.183 detected in the 12 survival patients, although the *p* value was over 0.05. This may be due to insufficient samples and short follow-up. Taken together, miR-122 is expected to become an effective indicator for predicting the survival rate of liver cancer patients.

RETRACTED

As the sample size was limited, the effects of miR-122 in chronic HBV patients have to be assessed in larger cohorts involving cases in diverse phases.

## 5. Conclusion

This study revealed that miR-122 could be utilized to screen patients with CHB infection. The peak level of serum miR-122 was found in CHB patients, with the progression of hepatitis B and serum miR-122 levels decreased gradually, providing novel insights into the mechanism of HBV-triggered illnesses. Overall, miR-122 is associated with hepatitis B activity, liver cell damage, and liver disease progression. It participates in the whole process of CHB and is anticipated to be a molecular marker for predicting the progression of CHB.

## Figures and Tables

**Figure 1:** Serum miR-122 expression in each group.

**Figure 2:** (a) Detection of miR-122 in CHB. (b) Correlation between miR-122 and albumin.

**Figure 3:** (a) miR-122 expression with Child-Pugh. (b) Correlation between miR-122 and HVPG. (c) miR-122 expression in HVPG ≤ 10 mmHg and HVPG > 10 mmHg.

**Figure 4:** (a) Correlation between miR-122 and AKP. (b) Correlation between miR-122 and AFP.

**Table 1:** Clinical data of four groups in study subjects.

Clinical data	Healthy (*N* = 10)	CHB (*N* = 11)	Cirrhosis (*N* = 26)	HCC (*N* = 16)	*P* value
Age	61.5 ± 5.1	53.1 ± 3	59.1 ± 2.5	62.3 ± 3.5	0.447
Male (%)	60	54.5	80.8	75	0.336
Hb	134.1 ± 26.71^a,b^	133.64 ± 16.11^c,d^	103.31 ± 31.24^a,c^	101.31 ± 30.19^b,d^	0.002
WBC	5.33 ± 1.49	6.29 ± 2.71	97.04 ± 60.59^a,c^	118.75 ± 65.65^b,d^	≤0.01
PLT	195.89 ± 90.51^a,b^	211.64 ± 79.08^c,d^	4.31 ± 2.03	5.96 ± 4.25	0.158
Ur	6.41 ± 4.71	4.75 ± 1.23	5.98 ± 2.41	8.23 ± 5.29	0.092
Cr	80.44 ± 33.33	71.00 ± 17.47	71.54 ± 14.54	101.25 ± 54.27	0.032
AST	33.10 ± 26.43	163.00 ± 315.03	40.96 ± 25.22	150.86 ± 225.52	0.081
ALT	27.22 ± 25.03	211.73 ± 407.64	34.73 ± 38.92	100.38 ± 168.27	0.068
TB	14.51 ± 7.49^a^	13.12 ± 8.15^b^	27.32 ± 16.59^a,b^	50.28 ± 56.77	0.010
DB	5.86 ± 3.32^a^	7.00 ± 5.23^b^	14.74 ± 11.54^a,b^	30.68 ± 40.11	0.017
AKP	85.67 ± 52.38	73.55 ± 36.53	83.50 ± 37.63	162.56 ± 130.3	0.050
Alb	44.67 ± 4.39	36.36 ± 4.55	35.42 ± 7.08	29.50 ± 7.23	≤0.01
AFP	2.49 ± 1.51	40.96 ± 72.78	9.56 ± 15.59	610.48 ± 591.12	≤0.01

Data are mean ± SD. CHB, chronic hepatitis B; HCC, hepatocellular carcinoma; WBC, white blood cell; PLT, platelet; Ur, urea; Cr, creatinine; AST, aspartate aminotransferase; ALT, alanine aminotransferase; TB, total bilirubin; DB, direct bilirubin; AKP, alkaline phosphatase; Alb, albumin; AFP, alpha-fetoprotein; ^a^, ^b^, ^c^_,_ and ^d^: *P* < 0.05, significant between-group differences.

RETRACTED

## Data Availability

The data used to support the findings of this study are available from the corresponding author upon request.

## Abbreviations

HBV: Hepatitis B virus
CHB: Chronic hepatitis B
HCC: Hepatocellular carcinoma
ALT: Alanine aminotransferase
AST: Aspartate aminotransferase
AKP: Alkaline phosphatase
miRNAs: MicroRNAs
HVPG: Hepatic venous pressure gradient
miR-122: MicroRNA-122
ncRNAs: Non-coding RNAs
BP: Biological processes
HCV: Hepatitis C virus
AIH: Autoimmune hepatitis
HGB: Hemoglobin
AFP: Alpha-fetoprotein
CSPH: Clinically significant portal hypertension.
